# Analysis of Adverse Reactions of Aspirin in Prophylaxis Medication Based on FAERS Database

**DOI:** 10.1155/2022/7882277

**Published:** 2022-05-26

**Authors:** Weidong Ren, Weihua Wang, Yanli Guo

**Affiliations:** ^1^Department of Neurosurgery, Mengyin People's Hospital, Linyi City 276200, Shandong Province, China; ^2^Pharmacy Department, Chengyang People's Hospital, Qingdao City 266000, Shandong Province, China; ^3^Department of Neurology, Jinnan Nanjiao Hospital, Jinan City 250000, Shandong Province, China

## Abstract

**Objective:**

As the most commonly used drug in the world, aspirin has shown benefits for myocardial infarction, stroke, and vascular death in many secondary prevention trials and their meta-analysis. The purpose of this study was to evaluate the association between aspirin and its adverse reactions as a preventive drug using the FDA adverse event reporting system (FAERS).

**Methods:**

The FAERS database was queried for the adverse drug events (ADE) reported from the first quarter of 2004 to the second quarter of 2021. We counted and trended reports to FAERS in which aspirin was associated with anaphylaxis or anaphylaxis followed by death.

**Results:**

The search retrieved 858 aspirin-associated cases within the reporting period; 108 AE pairs with significant disproportionality were retained. The top 10 AE pairs associated with using aspirin for prophylaxis were melaena, duodenal ulcer, gastritis erosive, gastric ulcer hemorrhage, etc. The top 10 AE pairs for thrombosis prophylaxis were melaena, duodenal ulcer, microcytic anemia, lip erosion, vascular stent thrombosis, etc. The screened adverse event reports are classified and counted according to the system organ class (SOC); it mainly focuses on gastrointestinal disorders, general disorders, and administration site conditions. Among the 858 cases of aspirin used as prophylaxis medication in the FAERS database, the reporting areas were mainly in Europe and the Americas.

**Conclusion:**

Adverse drug reactions may occur in the clinical use of aspirin. It should strengthen patient medication education, pay close attention to adverse reactions, and adjust the administration method in time to ensure the safety of medication.

## 1. Introduction

Aspirin (acetylsalicylic acid (ASA)) is the most commonly used drug in the world, and its use is fundamental for the prevention and treatment of cardiovascular diseases, especially acute coronary syndrome (ACS) and chronic ischemic heart disease (CIHD), as well as cerebrovascular diseases and some chronic rheumatic diseases [1, 2]. Antiplatelet agents are often used in the secondary prevention of ischemic stroke [3, 4]. As the earliest and most widely used antiplatelet agent in clinic, aspirin is usually used as the first choice in China. However, it has some risks and limitations in clinical treatment because of its adverse reactions such as gastrointestinal reaction, bleeding, and aspirin resistance [5, 6]. Therefore, any further data generated from the “real-life” repository or/and a unified national registry is particularly useful.

The FDA adverse event reporting system (FAERS) is a database designed to support FDA's postmarketing monitoring plan for drugs and therapeutic biological products [7]. The database includes all adverse drug event (ADE) information and mismedication information collected by FDA [8]. Because of its large amount of data, diverse data information, and free access to the public, it is often used in the research of ADE signal mining [9]. The FAERS database receives about 1.5 million ADE information reports on drugs and medical devices from the real world every year. These reports are spontaneously reported by professionals such as drug manufacturers, hospital medical staff, pharmacists, and pharmaceutical manufacturer staff, as well as patients, patient families, and lawyers [10].

To the best of our knowledge, there are no studies using the FAERS database to compare the association between aspirin and secondary stroke prevention. This study analyzes the adverse event information of aspirin collected in the FAERS database and excavates the potential adverse events of aspirin in secondary stroke prevention, in order to provide reference for optimizing patients' treatment plan, preventing, and coping with adverse drug reactions.

## 2. Material and Methods

### 2.1. Data Source

A retrospective pharmacovigilance study was performed using data from the FAERS database covering the period from the first quarter of 2004 to the second quarter of 2021. FAERS is a spontaneous reporting system (SRS) that contains adverse event reports, medication error reports, and product quality complaints resulting in adverse events submitted to FDA by healthcare professionals, consumers, manufacturers, and patients. The database contains demographic information, drug information, and reaction information. Each report has a primary suspected drug with one or more adverse drug reactions (ADR) and may include other drugs taken by the patient.

### 2.2. Data Mining

FAERS data requires substantial curate cleaning and normalizing before they can be used appropriately; otherwise, data can have a material impact on analysis results. Python (version 3.8) and PostgreSQL (version 12) are used to deal with the cleaning and normalization process, including merging data, deleting duplicate records, applying standardized vocabulary and drug names mapped to RxNorm concept and indications and results mapped to SNOMED-CT concept, standardizing the response to MedDRA (version 24.0) concept, and using R software (version 4.1.0) to statistically calculate drug response signals.  Figure 1 presents the main steps.

### 2.3. Statistical Analysis

Select “aspirin” as the drug name and report the role code as “ps-ss” (primary suspect and secondary suspect drugs) and indication with the prophylaxis from DRUG_INDI to be evaluated. In total, 4237 adverse events (AEs) paired were retrieved.

Both disproportionality analysis and *Bayesian* analysis applied with the use of the proportional reporting ratio (PRR), Bayesian confidence propagation neural network (BCPNN), and multi-item gamma Poisson shrinker (MGPS) were algorithms to investigate the potential signals between the drug and the specific adverse event of interest. The equations and criteria for the four algorithms above are demonstrated in Table 1. One of the four algorithms that meet the criteria should be considered a positive signal.

### 2.4. Compliance with Ethics Guidelines

All procedures performed in this study involving human participants were in accordance with the 1964 Helsinki declaration.

## 3. Results

During the study period (from the first quarter of 2004 to the second quarter of 2021), a total of 3,422,047 reports were submitted to FAERS. In total, 4237 AE paired reports of aspirin were reported, and 858 cases of reports have been found. Of these events, the top five indications for aspirin prophylaxis are prophylaxis (48%), thrombosis prophylaxis (38%), cardiovascular event prophylaxis (5%), cerebrovascular accident prophylaxis (4%), and ischemic heart disease prophylaxis (4%) (Figure 2), which is roughly consistent with the clinical medication.

In Table 2, when aspirin is used as thrombosis prophylaxis, the adverse reactions mostly occurred 1~9 months after the medication, and most of them occurred at 3~6 months. When aspirin is used as prophylaxis, the number of adverse reactions is mostly after 12 months, and the number of adverse reactions that occurred in 12~24 months, 24~60 months, and 60~ months was basically the same. When aspirin is used as cardiovascular event prophylaxis, ischemic heart disease prophylaxis, and cerebrovascular accident prophylaxis, there is no difference in the number of adverse reaction times (Table 2).

After analysis, we got 108 AE pairs with positive signals for a total of 858 cases. The top 10 in the number of adverse event reports associated with using aspirin for prophylaxis from the FAERS database were melaena, duodenal ulcer, gastritis erosive, gastric ulcer hemorrhage, blood loss anemia, duodenal ulcer hemorrhage, dyspnoea at rest, urinary tract discomfort, erosive duodenitis, and naevus flammeus (Table 3). The top 10 in the number of adverse event reports associated with using aspirin for thrombosis prophylaxis were melaena, duodenal ulcer, microcytic anemia, lip erosion, vascular stent thrombosis, mucosal erosion, Nikolsky's sign, hematoma muscle, vascular stent stenosis, and thalamus hemorrhage (Table 4). Among the top 10 adverse event reports, there are many similarities (melaena and duodenal ulcer) between the application of aspirin in prophylaxis and thrombosis prophylaxis.

The screened adverse event reports are classified and counted according to the system organ class (SOC); it can be seen from Table 5 that aspirin involves in 21 systems, mainly focusing on gastrointestinal disorders (63.2%); general disorders and administration site conditions (6.6%); blood and lymphatic system disorders (4.5%); injury, poisoning, and procedural complications (3.8%); skin and subcutaneous tissue disorders (3.7%); etc.

The clinical characteristics of events with aspirin are described in Table 6. The majority of adverse events came from Europe (552 (64.34%)) and the Americas (188 (21.91%)). The main sources of reports were physician (29.6%), other health professional (28.3%), consumer (20.7%), and pharmacist (16.1%). Of these events, 45.9% occurred in female, 46.7% occurred in male, and 7.3% of the events were gender unknown (Table 6). The proportion of males and females in 858 cases is balanced, consistent with the results of previous studies, and there is no obvious gender difference. The adverse reactions of aspirin had a peak in 2015-2016, then decreased slightly, and then formed a growth peak in 2018-2019. After that, the number of adverse events decreased significantly. This trend was also reflected in the change of the number observed by year in the following clinical characteristics in Table 6. Patients were mainly aged >65 years, which was numerically older than the median age of patients typically enrolled in clinical trials. The therapy duration groups in different months were similar. As shown in Table 7, the outcome most occurred as hospitalization or other serious important medical event in the prophylaxis and thrombosis prophylaxis indications of aspirin. Death or life-threatening events often occurred, respectively.

## 4. Discussion

Aspirin is a kind of salicylic acid derivative, which is mainly used to relieve pain and fever in clinic. In addition, with the increase of research, it is found that aspirin also has a good antiplatelet aggregation effect and has good curative effects on preventing postoperative thrombosis, myocardial infarction, transient ischemic attack, and angina pectoris [11]. After a lot of clinical observation, the role of aspirin in the primary prevention of cardiovascular disease (CVD) has been recognized; long-term adherence to aspirin can reduce the recurrence of cardiovascular events by 25%. The results of randomized controlled trials and meta-analysis show that high and low doses of aspirin have similar effects on the prevention of vascular events, but the risk of gastrointestinal bleeding is higher with higher doses of aspirin [12]. Therefore, the prevention of cardiovascular events with low-dose aspirin has been paid attention to and applied in clinical practice. The meta-analysis of the antithrombotic therapy collaborative group (ATC) in 2002 showed that 75~150 mg/d is the best dose for long-term use [1]. A large-scale clinical trial initiated by Chinese and British scientists and participated in nearly 1000 hospitals in 37 countries has confirmed that aspirin has a positive effect on ischemic stroke (cerebral ischemic stroke, CIS), which makes aspirin a proven effective and widely used drug in the treatment of ischemic stroke. This result shows that if aspirin is used for 2~4 weeks during the attack period, the mortality or stroke recurrence rate can be reduced by 11%. However, with the increase of clinical application and wide range of use of aspirin, the incidence of adverse reactions is also increasing [13]. How to reduce the incidence of adverse reactions while ensuring the effect of drug treatment has become a key problem in clinical practice.

Aspirin is initially used in antipyretic, analgesic, and anti-inflammatory. With the extensive research of scientists on their pharmacological effects, aspirin has been found to be effective in the treatment of rheumatic diseases, cardiocerebral vascular diseases, and diabetes [14]. In this study, we focused on the adverse effects of aspirin as a prophylaxis medication. From the results of this study, it is found that the top five indications for aspirin prophylaxis are prophylaxis, thrombosis prophylaxis, cardiovascular event prophylaxis, cerebrovascular accident prophylaxis, and ischemic heart disease prophylaxis, which is roughly consistent with the clinical medication. Arterial intravascular thrombosis leads to severe hypoperfusion and ischemia and hypoxia of tissues and organs, which is the root of cardiovascular, cerebrovascular, and peripheral arterial diseases. Thromboxane synthase A2 (TXA-2) and COX play an important role in thrombosis. Low-dose aspirin irreversibly combines with cyclooxygenase-2 (COX-2) to acetylate and inactivate it, so as to inhibit the formation of TXA-2, block TXA-2-mediated platelet aggregation, and inhibit thrombosis.

Aspirin has a wide range of clinical applications and good effects, but in the process of medication, it can lead to a variety of adverse reactions, mainly involving the respiratory system, digestive system, blood system, urinary system, etc. [15]. Aspirin can not only inhibit platelet cyclooxygenase and reduce the production of prostaglandin (PG) but also directly destroy the hydrophobic protective barrier of gastric mucosa, resulting in mucosal damage. Long-term use of aspirin to prevent thrombosis will increase the probability of adverse drug reactions, and adverse events will increase over time. Gastrointestinal reactions are the most common adverse reactions in the clinical application of aspirin, which is also confirmed by the results of this study. Long-term aspirin use increases the risk of gastrointestinal mucosal injury and is dose-related. Low-dose aspirin 10 mg/d can inhibit PG synthesis and cause damage to gastrointestinal mucosa. Aspirin 100 mg/d can increase the incidence of gastrointestinal bleeding by 1.5 times [16] and the incidence of asymptomatic gastrointestinal injury by 4 times [17]. Domestic studies have found that the incidence of gastrointestinal ulcer in patients taking aspirin is 4.79%, of which the incidence of upper gastrointestinal bleeding (UGIB) is 5.30%, and the relative risk of gastrointestinal perforation even reaches 6.64% [18]. There is a total of 9 randomized clinical trials of long-term oral aspirin for primary prevention of cardiovascular and cerebrovascular diseases. Meta-analysis showed that the risk of gastrointestinal bleeding increased by 1.37 times [19]. The mortality of lower gastrointestinal bleeding (LGIB) is higher. Common adverse reactions to aspirin are mainly gastrointestinal disorders, among which nausea, vomiting, upper abdominal discomfort, or pain is more common; long-term or large doses can cause gastrointestinal bleeding or ulcers, but severe gastrointestinal bleeding is rare.

From the results of the article, we can find that the number of adverse reactions to aspirin has a peak from 2015 to 2016 and then a higher peak from 2018 to 2019, which may be due to changes in some guidelines during this period (US Preventive Services Task Force (USPSTF 2016), American Diabetes Association (ADA 2019), American College of Cardiology and American Heart Association (ACC/AHA 2019), and European Society of Cardiology (ESC 2016)). For example, aspirin should not be used for the primary prevention of cardiovascular disease [20], whereas others have suggested that aspirin is offered to individuals in a certain age range and/or above some given level of predicted risk of cardiovascular disease [21, 22]. Uncertainty on aspirin use has been reflected in current guideline recommendations [23, 24], and aspirin use for primary prevention has been controversial even when compared with aspirin use in patients with established atherosclerotic cardiovascular disease.

Studies have shown that age is an important risk factor for aspirin-related bleeding; the bleeding risk of elderly patients after aspirin application is significantly increased [25], which seriously affects the benefit of aspirin in reducing cardiovascular events. The Japanese primary prevention study published in JAMA in 2014 showed that the treatment of 14464 elderly patients aged 60~85 with aspirin (100 mg/d) significantly increased the risk of extracranial hemorrhage and did not reduce the combined endpoint including death [26]. Therefore, for elderly patients, especially elderly patients, the use of aspirin needs to weigh the cardiovascular benefit and bleeding risk, adhere to the principle of individualized treatment, minimize bleeding complications, and enable them to benefit from aspirin treatment.

Further excavation of the FAERS database can expand new ideas for evaluating the safety of drugs and is a research method that is worthy of further in-depth development. But this method also has limitations. Firstly, because FAERS data is a voluntary report, including public reports; there are problems such as underreporting, selective reporting, and lack of information. Secondly, although the analysis shows that there is a statistical correlation between the drug and the adverse event, the actual causality still needs further verification. In addition, most of the FAERS data come from European and American populations and relatively few Asian populations.

In conclusion, this study used the FAERS database to propose the safety signal between the use of aspirin and the clinical prevention of adverse events. Since this study is based on a spontaneous reporting database that inevitably contains potential deviations, cohort studies and long-term data are still needed to verify these results and further understand the safety of aspirin.

## Figures and Tables

**Figure 1:** Main steps of process.

**Figure 2:** Indication of using aspirin for prophylaxis.

**Table 1:** Summary of major algorithms and criteria used for signal detection.

Algorithms	Equation	Criteria
ROR	ROR=*ad*/*bc*	ROR ≥ 1, CI025 ≥ 1
	$95\%\text{CI}=e^{\ln\left(\text{ROR}\right)\pm 1.96\sqrt{\left(1/a+1/b+1/c+1/d\right)}}$	

PRR	PRR=*a*(*c* + *d*)/*c*(*a* + *b*)	PRR ≥ 2, *χ*^2^ ≥ 4, *a* ≥ 3
	$95\%\text{CI}=e^{\ln\left(\text{PRR}\right)\pm 1.96\sqrt{1/a-1/\left(a+b\right)+1/c+1/\left(c+d\right)}}$	
	$\chi^{2}=\sum \frac{{\left(O-E\right)}^{2}}{E}\;\left(O=a,E=\frac{\left(a+b\right)\left(a+c\right)}{a+b+c+d}\right)$	

BCPNN	IC = log_2_*a*(*a* + *b* + *c* + *d*)(*a* + *c*)(*a* + *b*)	IC25‐2sd > 0
	$95\%\text{CI}=e^{\ln\left(\text{IC}\right)\pm 1.96\sqrt{1/a+1/b+1/c+1/d}}$	

MGPS	$\text{EBGM}=\frac{a\left(a+b+c+d\right)\left(a+b\right)}{a+c}$	EBGM05 ≥ 2

**Table 2:** Changes in the number of adverse reactions after aspirin administration with different medication indications with medication time.

Indications	0~1 month	1~3 months	3~6 months	6~9 months	9~12 months	12~24 months	24~60 months	60~ months	Total	Average (day)	Average (day)	std dev
Thrombosis prophylaxis	19	35	53	37	26	20	18	8	216	471.0		
Prophylaxis	21	12	15	10	6	34	33	43	174	1324.8		
Cardiovascular event prophylaxis	1	5	0	1	0	1	1	5	14	1637.6	871.1	1498.9
Ischemic heart disease prophylaxis	2	0	2	0	0	0	1	1	6	606.7		
Cerebrovascular accident prophylaxis	2	0	1	0	0	0	2	0	5	538.2		

**Table 3:** The top 10 adverse event reports associated with using aspirin for prophylaxis from the FAERS database (January 2004 to June 2021).

Reactions	Indication	*n*	ROR (95% CI)	PRR (95% CI, *χ*^2^)	BCPNN (IC-2SD)	EBGM (EBGM05)
Melaena	Prophylaxis	101	1.55 (1.28, 1.89)	1.55 (1.35, 1.75, 19.08)	0.62 (0.6)	1.55 (1.38)
Duodenal ulcer	Prophylaxis	48	2.29 (1.72, 3.04)	2.29 (2.01, 2.57, 33.38)	1.15 (1.11)	2.28 (2.04)
Gastritis erosive	Prophylaxis	46	3.29 (2.46, 4.4)	3.29 (3, 3.58, 70.1)	1.64 (1.59)	3.26 (3.02)
Gastric ulcer hemorrhage	Prophylaxis	42	2.29 (1.69, 3.11)	2.29 (1.99, 2.6, 29.16)	1.15 (1.11)	2.28 (2.03)
Blood loss anemia	Prophylaxis	33	1.54 (1.09, 2.16)	1.54 (1.2, 1.88, 5.63)	0.59 (0.56)	1.53 (1.25)
Duodenal ulcer hemorrhage	Prophylaxis	21	2.06 (1.34, 3.16)	2.06 (1.63, 2.49, 10.29)	0.97 (0.91)	2.05 (1.69)
Dyspnoea at rest	Prophylaxis	13	1.78 (1.03, 3.07)	1.78 (1.24, 2.33, 3.69)	0.75 (0.69)	1.78 (1.32)
Urinary tract discomfort	Prophylaxis	9	13.46 (6.9, 26.25)	13.46 (12.79, 14.13, 87.65)	2.56 (2.35)	12.91 (12.35)
Erosive duodenitis	Prophylaxis	7	2.43 (1.15, 5.1)	2.43 (1.68, 3.17, 4.48)	1.04 (0.94)	2.41 (1.79)
Naevus flammeus	Prophylaxis	5	8.1 (3.33, 19.69)	8.1 (7.21, 8.99, 23.73)	1.87 (1.66)	7.91 (7.16)
Total		325				

**Table 4:** The top 10 adverse event reports associated with using aspirin for thrombosis prophylaxis from the FAERS database (January 2004 to June 2021).

Reactions	Indication	*n*	ROR (95% CI)	PRR (95% CI, *χ*^2^)	BCPNN (IC-2SD)	EBGM (EBGM05)
Melaena	Thrombosis prophylaxis	127	1.95 (1.64, 2.33)	1.95 (1.78, 2.13, 57.64)	0.95 (0.93)	1.95 (1.8)
Duodenal ulcer	Thrombosis prophylaxis	31	1.48 (1.04, 2.1)	1.48 (1.12, 1.83, 4.26)	0.54 (0.5)	1.47 (1.18)
Microcytic anemia	Thrombosis prophylaxis	25	3.59 (2.42, 5.32)	3.58 (3.19, 3.98, 43.51)	1.69 (1.63)	3.55 (3.22)
Lip erosion	Thrombosis prophylaxis	22	3.85 (2.53, 5.86)	3.85 (3.42, 4.27, 42.94)	1.76 (1.69)	3.81 (3.46)
Vascular stent thrombosis	Thrombosis prophylaxis	22	3.99 (2.62, 6.07)	3.99 (3.57, 4.41, 45.67)	1.81 (1.73)	3.95 (3.6)
Mucosal erosion	Thrombosis prophylaxis	21	3.86 (2.51, 5.94)	3.86 (3.43, 4.29, 41.12)	1.76 (1.69)	3.82 (3.46)
Nikolsky's sign	Thrombosis prophylaxis	18	4.02 (2.53, 6.41)	4.02 (3.56, 4.49, 37.42)	1.78 (1.7)	3.98 (3.59)
Hematoma muscle	Thrombosis prophylaxis	16	8.02 (4.88, 13.17)	8.02 (7.52, 8.51, 88.91)	2.48 (2.36)	7.83 (7.41)
Vascular stent stenosis	Thrombosis prophylaxis	8	3.58 (1.78, 7.19)	3.58 (2.88, 4.28, 12.25)	1.47 (1.35)	3.55 (2.97)
Thalamus hemorrhage	Thrombosis prophylaxis	8	3.13 (1.56, 6.28)	3.13 (2.43, 3.83, 9.46)	1.33 (1.23)	3.11 (2.53)
Total		298				

**Table 5:** AEs of aspirin at the system organ class (SOC) level in FAERS database.

System organ class (SOC)	Cases reporting (*n* = 858)	
Gastrointestinal disorders	542	63.2%
General disorders and administration site conditions	57	6.6%
Blood and lymphatic system disorders	39	4.5%
Injury, poisoning, and procedural complications	33	3.8%
Skin and subcutaneous tissue disorders	32	3.7%
Cardiac disorders	26	3.0%
Investigations	25	2.9%
Renal and urinary disorders	23	2.7%
Musculoskeletal and connective tissue disorders	18	2.1%
Respiratory, thoracic, and mediastinal disorders	17	2.0%
Nervous system disorders	16	1.9%
Vascular disorders	14	1.6%
Infections and infestations	10	1.2%
Neoplasms benign, malignant, and unspecified (incl cysts and polyps)	6	0.7%
Metabolism and nutrition disorders	5	0.6%
Reproductive system and breast disorders	5	0.6%
Eye disorders	2	0.2%
Endocrine disorders	1	0.1%
Surgical and medical procedures	1	0.1%
Psychiatric disorders	1	0.1%
Social circumstances	1	0.1%

**Table 6:** Clinical characteristics of patients with adverse reactions to aspirin collected from the FAERS database.

Characteristics	Report no.	%
*Reporting region*		
Europe	552	64.34%
Oceania	3	0.35%
Americas	188	21.91%
Asia	76	8.86%
Africa	4	0.47%
Unknown or missing	35	4.08%
*Reporters*		
Consumer	178	20.7%
Other health professional	243	28.3%
Pharmacist	138	16.1%
Physician	254	29.6%
Unknown	45	5.2%
*Reported year*		
2004 and before	26	3.0%
2005	34	4.0%
2006	13	1.5%
2007	4	0.5%
2008	12	1.4%
2009	7	0.8%
2010	8	0.9%
2011	23	2.7%
2012	18	2.1%
2013	43	5.0%
2014	58	6.8%
2015	95	11.1%
2016	92	10.7%
2017	72	8.4%
2018	141	16.4%
2019	119	13.9%
2020	66	7.7%
2021Q1Q2	27	3.1%
*Gender*		
Female	394	45.9%
Male	401	46.7%
Unknown	63	7.3%
*Age group*		
0 to 18	5	0.6%
18 to 45	83	9.7%
45 to 65	93	10.8%
65 to 75	238	27.7%
75 to	342	39.9%
Unknown	97	11.3%
*Therapy duration groups*		
0~1 month	45	5.24%
1~3 months	52	6.06%
3~6 months	71	8.28%
6~9 months	48	5.59%
9~12 months	32	3.73%
12~24 months	55	6.41%
24~60 months	55	6.41%
60~ months	57	6.64%
Unknown	443	51.63%

**Table 7:** Outcome of patients after adverse reactions of aspirin under different indications.

Indications	Hospitalization—initial or prolonged	Other serious (important medical event)	Death	Life-threatening	Disability	Required intervention to prevent permanent impairment/damage
Prophylaxis (NEC)	350	228	19	26	0	2
Thrombosis prophylaxis	231	148	95	53	6	3
Cardiovascular event prophylaxis	13	21	2	21	6	0
Ischemic heart disease prophylaxis	14	34	1	7	1	0
Cerebrovascular accident prophylaxis	37	14	4	0	1	0
Blood disorder prophylaxis	8	8	0	6	0	0
Prophylaxis of abortion	1	2	0	1	1	0
Atherosclerosis prophylaxis	1	1	1	0	0	0
Renal disorder prophylaxis	0	1	0	0	0	0
Total (%)	655	457	122	114	15	5
Therapy durations	1024.9	1212.3	365.2	447.4	877.8	580.3

## Data Availability

The datasets used and/or analyzed during the present study are available from the corresponding author on reasonable request.
